The article "The perception of Hungarian food by consumer segments according to food purchasing preferences based on primary research results" was retracted in 2025. Reasons: concerns about the data; concerns about the results or conclusions.

# The perception of Hungarian food by consumer segments according to food purchasing preferences based on primary research results

**DOI:** 10.1371/journal.pone.0273023

**Published:** 2022-08-24

**Authors:** Mónika Garai-Fodor, Anett Popovics, Ágnes Csiszárik-Kocsir

**Affiliations:** Keleti Károly Faculty of Business and Management, Óbuda University, Budapest, Hungary; Hungarian University of Agriculture and Life Sciences: Magyar Agrar- es Elettudomanyi Egyetem, HUNGARY

## Abstract

In addition to the intrinsic value of the product, social, cultural and psychological factors also have a major influence on the consumer’s purchasing decision. They are also influenced by trends and tendencies such as globalisation, digitalisation and various economic and social crises. In our study, we focused on the analysis of food purchasing preferences; including the reasons for the rise of ethnocentrism in the purchase of domestic products and the potential of this phenomenon in light of relevant secondary data and quantitative primary results. The main objective of the study’s primary research is to demonstrate that consumer groups, distinguishable by food consumption preferences, have differentiated perceptions of domestic food (price, quality, reliability). This provides evidence that food consumer preferences are reflected in decisions about domestic food. Due to the Hungarian relevance of the topic, the presentation of related international research and literature was given a prominent role. The focus of our research was to investigate the food purchasing preferences of Hungarian food consumers. Based on the results, we were able to characterise distinct consumer segments based on food purchasing preferences, and we were able to identify potential target groups of domestic food based on food consumer preferences: the ‘conscious food buyers’, the ‘impulse buyers’ and the ‘no preference’. In our view, members belonging to the first two segments can be successfully persuaded to buy Hungarian food through an educational campaign based on sufficiently fashionable and trendy motifs with the help of the right reference person.

## Introduction

Food plays a central role in people’s lives. The proportion spent on food is the highest among consumer expenditures and the most time spent on average per year on food. Food consumption is both a compulsion and a source of pleasure, it determines the lifestyle and rhythm of consumers, their social relationships and can be traced back to the traditions of particular cultures. According to Lehota [1], the factors that influence food consumption behaviour are: biological, psychological, sociological, anthropological, demographic, economic and political. A cardinal issue in consumer behaviour is the study of consumer attitudes and the patterns of behaviour that emerge from them. There is a trend in consumer behaviour towards seeing food as a cultural phenomenon rather than simply an agricultural product. According to Sini [2], this occurs when the product is associated with a specific use, a tradition, or when it is acquired in a specific place. The interest in products linked to culture and place can open up market niches, creating the opposite of the standardisation of consumption [3]. The observation of consumer behaviour and attitudes is always a novel field that can never be fully explored, but it can identify trends and influences that override previous findings.

In this study, we focus on the cultural determinants of food consumption behaviour, as emphasised in the literature. The research will focus on the impact of food origin, including its regional affiliations, on consumer preferences. In this sense, the theoretical basis of the study is formed by those approaches to food consumption that make greater emphasis on the influential role of anthropological factors alongside biological, psychological and sociological aspects.

In this study, we focus on secondary sources of domestic food consumption behaviour, given that our primary research also seeks to answer the question of what food consumption preferences characterise domestic food consumers. We consider a product to be a domestic food if more than 50% of the ingredients used are Hungarian and each step of the production process takes place in Hungary. A Hungarian product is defined as a product made from 100% Hungarian ingredients [1].

## Literature review

### Trends in food consumer preferences

Based on the main objective of the study, the literature review aimed to cover food consumer research, with a special focus on studies related to domestic food. Food has the greatest share of consumer spending and, on an annual basis, consumers devote the majority of their time to buying food. Food consumption is both a necessity and a source of pleasure; it influences consumers’ lifestyles and rhythms as well as their social relationships, and can be traced back to cultural traditions. According to Lehota [1], factors influencing food consumer behaviour include the following: biological, psychological, sociological, anthropological, demographic, economic, and political factors.

The study of consumer attitudes and the resulting patterns of behaviour is a crucial aspect of consumer behaviour [4–8]. Food, rather than being viewed as a straightforward agricultural product, is increasingly being understood as a cultural moment in consumer behaviour. According to Sini [2], this happens when a product is tied to a particular use, tradition, or is bought at a unique place. Interest in culturally and locally based goods will create market niches, reversing the trend of consumer standardization [3]. Observing consumer behaviour is often an area that conceals novelties that can never be completely understood, but it can reveal directions and effects that overpower previous facts [9]. We are currently seeing changes that are primarily aimed at self-realization and self-expression, diverging from the previously-held conventional value system. Recent food research has revealed a consumer need for sustainability and the significance of the concept of sustainability [10, 11]. A majority of customers embrace sustainability as a value, but this is not always the case in their behaviour as proven by many authors [12, 13]. This is also true for food consumption as evidenced by many studies [14]. The 2008 financial crisis, a milestone in consumer history, completely rewrote the rules. Nowadays, the consumer ‘is breathing’ again after the tight time which was followed by a recovery, but it should be noted that with the current coronavirus crisis, we are approaching another stage in terms of consumption trends. Törőcsik [15] writes about a predictable, unpredictable, reasoned, and crisis-stricken consumer in connection with the phenomenon and, in a later writing [16], trends such as delay, non-purchase, or mystery shopping are identified.

Variety, dynamism, and volatility are all essential aspects of a consumer market; resulting in unpredictability. Globalization [17] and digitalization [18] have a significant impact on bolstering these factors, aided by the ongoing coronavirus outbreak. These consequences cause people to rethink their shopping habits which can be traced not only to the purchase of durable goods but also to the purchase of food. In today’s world, the ability to shop online is becoming increasingly relevant in the food market. The new and unprecedented situation has prompted new challenges and reactions from both retailers and wholesalers in the food market [19].

Törőcsik [20] distinguishes between the trend of experience-seeking and its opponent, i.e., the search for authenticity among consumer expectations. The provision of experience-like shopping conditions as well as consumer demand for attractions and show elements, has become a requirement in recent years. As the consumer is bombarded with increasingly extreme visual elements, providing the experience is becoming more and more specific. As a rejection of this artificial and shallow phenomenon, searching for authenticity is becoming more and more prevalent among consumer expectations and decision-making components. Selecting a genuine, knowledgeable, and trustworthy producer, trader, or service provider is accompanied by consciousness and dedication. All of this is especially noteworthy when it comes to online shopping where visual elements are even more pronounced in the experience [21], differing significantly in the perception of each generation. Numerous studies and articles have been written about each generation’s shopping habits. Generation Y is known for having considerable purchasing power and the ability to handle digital gadgets, so they use them effectively to support their purchasing decisions. Generation X also represents purchasing power, but they feel more comfortable in the offline space and better at online shopping than the Baby Boomer generation.

In contrast, the digital native Generation Z lives almost entirely in the digital world, but remains low in terms of purchasing power; they are more of a mystery shopper, representing only a small proportion of real purchasing power [22]. Members of younger age groups prefer to shop online where a wider range of choice is provided, enhancing the shopping experience [23]. Online shopping is often aided by the fact that customers can obtain information about a product easily and at a low cost which is critical in the age of digitization. It is important to note, however, that online shopping will never totally replace offline shopping because there will still be customers and buyers who prefer to physically experience the product’s basic features and enjoy the atmosphere created by personal shopping which is an important part of the shopping experience [24].

A discerning customer requires openness and security of purchase in addition to high quality and brand. According to Lewis and Bridger [25], trust is becoming increasingly important in today’s world and, in order to build it, credibility in the area of perceived risk must be built. The buying decision can be simplified if trust is built, and trust, in our opinion, can be gained through the use of origin and quality indicators. Szente et al. [26] investigated food consumer behaviour patterns and found health to be an exceptional trend as a significant social value that is expected to play a pivotal role in the coming years. Customers are expected to consider food quality, comfort and food safety as well as a healthier lifestyle, in addition to costs.

According to [27] research, the following trend correlations influence food choice. According to her findings, symbolic content is increasingly important in food consumption, and varied and newer food trends are emerging as a result of the faster pace of life as well as altered consumer expectations and lifestyles (Table 1). These novelties are either accepted or rejected by consumers in a variety of ways, resulting in the formation of characteristic consumer groups. In the primary research of our study, we focus on the morality factor group by analysing the preference for domestic products, partly touching on the lifestyle dimension related to values and the health trend group in terms of awareness.

**Table 1:** Food choice is influenced by the following trend correlations.

Body	Health	Morality	Experience	Lifestyle
show marketability control	science consciousness principles control experts	environmental consciousness sustainability fears ethical considerations responsibility	enjoy aesthetic vision fresh individuality indulgence mobility	apparent consumption self-expression luxury

Source: authors‘ own compilation based on Törőcsik [27]

In March 2020, during the first wave of coronavirus epidemic, Soós [28] examined food consumer habits through a questionnaire survey. According to the results, the role of smaller local shops and markets in the purchases of domestic consumers has increased in relation to supermarkets and hypermarkets. As local small-scale retailers often delivered food to their homes, personal contact became more important, and even confidence in local products and food increased. Previous experiences has greatly influenced the food choice, so the emphasis on trust has become a key message in brand communication during the epidemic.

Madarász [29] also examined the purchasing behavior of Hungarian consumers with his colleagues in the first wave of the epidemic. According to the results, the food choice motivations of Hungarian consumers did not change in the first wave of COVID-19; however, the order of preference has changed. During the period under review, the excellent taste of the products and the consistently high quality of the selected products maintained their leading position, overtaking, for example, health. The importance of the popular, familiar brand has diminished, suggesting that consumers are more likely to give up their regular brand if they experience a crisis. A further result of their survey is that consumer segments are basically divided into three parts; along with demanding and ethnocentric shoppers, taste preferences as well as rational shoppers were present. It is worth highlighting the demanding, quality-oriented shoppers, as they were the ones who lived extremely consciously during the quarantine period: they paid attention to food use, studied food labels more thoroughly, tried to eat healthier than before, and preferred local products.

Keller-Huszka [30] managed empirical research in the second wave of the Covid epidemic using quantitative methods. The aim of the study was to examine the changed consumer behavior of Hungarian consumers, especially the active population, middle-aged people and young people. According to their results, the demand for durable food has grown exponentially, and consumers have preferred discounts and local convenience stores. The increase in online food shopping is also clearly visible: food purchases were more conscious and cautious last year.

### Consumer behaviour on hungarian foods

Several consumer behaviour surveys have shown that ethnocentrism influences purchasing decisions and affects both product evaluation and buying intentions [31–36]. The consecutive ethnocentrism studies looked at buying intent and attitudes [31, 37–40]. Kim and Pysarchik [41] found a statistically significant negative correlation between consumer ethnocentrism and a desire to buy domestic products [42–45]. Ethnocentrism in consumption can be analysed from many angles and products, and has been the subject of numerous studies and research [8, 38, 46, 47].

This is possible, according to Moon and Nelson [48], because consumer behaviour is heavily influenced by cultural values, and this is so true in that consumers prefer domestically produced products as well as those from similar-cultured countries to products from other countries.

However, it is essential to emphasize that both economic growth and consumer welfare have an effect on ethnocentrism [32, 49]. Consumers in economically developed countries have a higher level of confidence in goods made in their own country, so ethnocentrism is stronger while consumers in less developed countries have a much lower level of confidence in products made in their own country [50].

As a result, it is critical to note that increased trust in domestic goods drives purchases. In fact, today’s consumers place a high value on food safety when shopping for food, expecting transparent information and quality assurances [51]. Buyers need to know everything there is to know about the product they buy [52]. However, it is very important to always keep in mind the issue of information reliability [53].

Non-ethnocentric consumers judge both domestic and foreign products on their quality while ethnocentric consumers rely more on country-of-origin information. Ethnocentric consumers consider purchasing products from abroad to be incorrect because it endangers the domestic economy. This effect is strongest when it comes to food purchases as customers develop a sense of nostalgia for emotional attachments to domestic food brands, and traditionally attribute good quality to these products [54]. In many cases, they do not feel a sense of attachment to foreign foods, and their sense of security is often lower than it is for domestic products since there are no guarantee components that would ensure traceability and recall [55].

Verlegh and Steenkamp [56] discovered that if the customer is confident enough that the product’s country of origin guarantees good quality, then ethnocentrism is demonstrably engaged in product assessment. Otherwise, before making a purchasing decision, the consumer examines each product feature individually.

To understand consumers’ motives, marketers must first understand their goals, product expertise, and attitude—all of which affect the decision-making process.

Ittersum [57] found that consumers had a more positive attitude toward goods from their own region after analyzing consumer target hierarchies in parallel with each step of the buying decision process. The findings show that the chance of a regional product being included in the buying decision depends to a large extent on how the consumer recognises it in the information seeking place. When a buying problem arises (internal information retrieval) or when the consumer encounters the product during the information retrieval phase, information about a regional product may be extracted from memory (external information retrieval). According to Ittersum [57], consumers are interested in the region and, therefore, the increasing interest may enhance the likelihood of encountering a regional product. Consumers’ attitudes and perception of regional products are often influenced by culture: the more consumers are drawn to a region’s culture, the more positive their attitudes toward regional products are.

Food consumption is part of socio-cultural status, according to Chaney’s [58] lifestyle model, so food and drink are also indicators of taste, fashion, and demandingness among lifestyle characteristics. Regional foods sometimes evoke nostalgia for the past when the consumer was younger or when they spent the vacations in good company [59]. Nostalgia for traditional flavors, village holidays and rural pastimes can especially be evoked among city dwellers. Individuals’ cultural identities are re-evaluated by local products, and these ideals and symbols contribute to the relocation of culture [60].

The final conclusions of a series of Hungarian research projects were in line with the international findings. Papadopoulos et al. concluded in 1990 [61] that the majority of Hungarians were not or only slightly ethnocentric. This is due to the fact that developing countries often raise the standard of living and goods of developed countries while underestimating the performance of their own countries. Hungarian products were normally devalued in Hungary at the time of the regime change as opposed to those from Western countries [62, 63].

Berács and Malota [64] found that Hungarian respondents were generally positive about domestic products ten years later, but that the perception of products from developed countries was still more favorable. Consumers still did not think domestic products were very good, according to a representative survey conducted later among the residents of Budapest [54], but, despite this, the desire to purchase Hungarian products was already the greatest.

Consumer habits and attitudes in the traditional Hungarian food market were studied by Szakály et al. [65]. According to the findings of the study, consumers interpret the term ‘classic Hungarian food’ to mean food prepared only with Hungarian flavors and following an old recipe. 97% of respondents consume some traditional Hungarian food; those who do not, cite high cost as a reason. Traditional food consumption is affected by the product’s flavor and consistent quality as well as family preferences and the quality guarantee offered via brand. Further study has shown that Hungarian food is consumed as part of daily meals and cannot be associated with a particular holiday or special occasion. Households with one or two people over the age of 40 and those in southern Hungary are more likely to consume traditional foods [66].

Several studies have looked at how people perceive food in the past and present alike. In terms of food quality, there is also evidence that consumers place a greater value on conventional foods than on foreign products. More than 40% of respondents believe that the quality of Hungarian food is superior to that of foreigners, and more than 80% believe that the quality of Hungarian food is good or excellent. Several studies have found that when purchasing food, Hungarian consumers prioritize the following factors: price, quality, healthiness, and Hungarian origin. Horváth et al. [67] investigated the impact of value systems on nutrition, identifying the basic dimensions of consumer behavioural trends as time, health, knowledge, credibility, and the desire for trust. As a result of their findings, they identified three groups of factors that reflect the Hungarian value system. The first group includes hedonistic values (independence, a lot of free time, an enjoyable life), the second group includes conventional values (family, balance, a peaceful life), and the third group includes financial security values (success, career, financial security). When it comes to basic foods, wellbeing, safety, a happy family life, and good human relations are the most important values for Hungarian consumers. Malota et al. [68] investigated the Hungarian population’s food purchasing and consumption preferences as well as eating habits. As a result of their research, six main groups were identified and their main criteria were as defined: ‘active maximalists’, ‘value-for-money seekers’, ‘like local specialties’, ‘everyday active’, ‘price-sensitive’, and ‘comfortable maximalists’. Of the 1,500 sample representative of the Hungarian population, one-fifth of respondents belong to the group of ‘those who like local specialties’. For these consumers, the image of the product is important, and for the food to be Hungarian, it must come from a local producer. Typically, respondents from central Hungary, young, with secondary or tertiary degrees, fall into this category and 58% are men.

Ferencz [69] examined the sales opportunities of local products and the consumer perception of local foods. The quantitative analysis showed that more and more buyers are looking for domestic, quality products. They know that the local economy is developing with the purchase of Hungarian products, but in many cases the price sensitivity of the Hungarian consumer comes to the fore. Internet already has the role of the largest information provider even in the case of traditional fairs and markets and that consumers prefer quality and a reliable source in their purchases–revealed from the research.

Further research has discovered that the market demand for Hungarian food products—according to the study traditional and regional meat products—is constantly growing. The target group of these products is loyal to the brand and has high quality expectations. In the case of local products, the guarantee of quality—the basis of branding—is typically the authenticity of the producer [70].

The growing interest in local food can be seen as a major trend in sustainable food consumption. Kovács [71] and colleagues examined the internal and external motivational factors of young consumers in a sample of 1756 respondents aged 18 to 45 years. According to their results, the characteristics related to local products include freshness, high quality, nutritional value, reliability, safety, recall of domestic flavors, naturalness, and healthiness. The main reason young people bought local food was taste and curiosity. Of the three groups formed by cluster analysis, the “value creators” segment considers local products to be healthy and nutritious.

The above results are also supported by the results of the representative survey of T. Nagy-Pető [72]. The respondents consider the identification of the place of origin, health and support of local producers to be the most important motivating factors. When it comes to where consumers can find information about local food, local producers can be considered as authentic sources.

## Material and method

The main research question of the present study is how different consumer groups perceive domestic food according to their food purchasing preference system: in terms of quality, price, reliability, motivation and reasons for purchasing.

Ethnocentric consumer behaviour refers to the positive perception and preference for domestic foods [65, 66]. We measured the consumption of domestic foods in our primary research; focusing on the manifestation of ethnocentrism in this consumer behaviour. The main objective of the quantitative research was to prove the relationship between food consumer preference and the perception of domestic food. Our aim was to create segments based on food buyer preference and to characterise them in terms of the perception of domestic food products: price, quality, the impact of domestic job creation, and to identify the motivations and influencing factors for their purchase.

The first stage of the research process was a systematic secondary source analysis. The study of food consumption is a central research topic in many disciplines. The secondary sources were used to outline the primary research phase which consisted of two phases: qualitative research as a pre-study and subsequent quantitative data collection. In the qualitative phase, 10 mini-focus group interviews were conducted using a semi-structured interview schedule. The main purpose of the qualitative research was to ground the quantitative research, pre-test the quantitative research tool and collect evidence for the questionnaire and hypotheses.

The qualitative research used a semi-structured interview design with the following topics: food purchasing habits, perceptions of domestic food retailers, characteristics, motivations and barriers to buying domestic food. The themes of the qualitative research guideline were determined by the results of the secondary source analysis and the purpose of the research. Qualitative sampling was carried out using the snowball method; firstly with the participation of the students themselves. The mini-focuses were conducted with 3–4 participants each with guided discussions in groups with a heterogeneous composition in terms of gender and age.

As a result of the qualitative phase, the themes of the quantitative research tool were developed and, subsequently, the specific questions were constructed, taking into account the results of the relevant secondary data analysis and the research objectives. The development and finalization of some response alternatives to the questionnaire—pre-testing of the quantitative research tool—was carried out in light of qualitative results. The second stage of the primary research was the quantitative phase, validating the qualitative results by exploring measurable outcomes. Quantitative data collection took the form of an online survey conducted using a pre-tested, standardized questionnaire. Subjects were recruited using a snowball sampling procedure, resulting in 1,447 evaluable questionnaires. Due to the sampling procedure of the research, the results cannot be considered representative, local, results for the sampling unit.

The research was made in the field of social sciences in online form. During the qualitative and quantitative research all participants were consent to participate (they could fill the form after agreeing only, based on the online rules). The online technology ensured the protection of privacy and anonymity. No race/ethnicity, age, disease/disabilities, religion, sex/gender, sexual orientation, or other socially constructed groupings related questions were raised. At our Faculty, there is no ethics committee to evaluate such research proposals, instead the Research Centre (headed by the Vice-Dean for Research of the Faculty and the members are the heads of the research teams) examines the circumstances of research. The research leaders have the supportive opinion of the research centre. Individuals participating in the research have been given a guarantee in the research description that their responses will be processed anonymously, without any identification. This fact was accepted when completing the questionnaire and the participants freely agreed to this. No children participated in the research.

The themes of the quantitative research tool were: food purchasing habits, food consumption preferences, domestic (Hungarian) food purchasing habits and domestic food consumption preferences, perceptions of Hungarian food (covering cognitive, affective and conative phases), and socio-demographic data. The research tool consisted of closed questions only, nominal—single- and multiple-choice selective questions—and four-point rating scales (4-point rating scale) for the analysis of consumer attitudes and value orientation. The scaling questions were based on a so-called coercive scale ranging from 1 to 4. One reason for this is the individual scale preference of Hungarian respondents: due to the school grading system, Hungarian respondents are most stable in interpreting the 5-point scale as opposed to the 1–7, 1–9 or 1–10 scales. And the even scale was chosen because the middle value (3) for the odd (1–5) scale is an escape route for respondents. In the analysis of attitudes, those who chose the middle value do not tip the scales in either direction, resulting in an excessive proportion of ‘indifferent’ consumers, making it difficult to segment them in a statistically and professionally meaningful way. We therefore opted for an even scale which, by excluding the middle value, gives the respondent a more rigorous stance, thus contributing more to a successful segmentation [73]. In addition, for the questions analysed using the odd-even scale, it was not necessary to have a middle, indifferent, value either as a ‘don’t know’ response as the cognitive level was filtered using separate questions. In this paper, we focus on the partial results of the quantitative phase of our research project. Within that, we have also focused on food purchasing habits, possible segmentation options based on preference, and the relationship of each food purchasing segment to Hungarian food.

## Objectives

The main hypotheses of the research were defined on the basis of the conclusions of the secondary data analyses and our own previous empirical experience.

We hypothesize that there is a relationship between food purchasing preferences and attitudes towards Hungarian food.

- Distinct consumer groups can be defined according to food consumer preferences (H1).
- There is a statistically verifiable correlation between the segments formed according to the preferences of food buyers and the attitude towards Hungarian food (H2).

In order to process the quantitative results and to test the hypotheses, we used descriptive statistics, bivariate and multivariate analyses using SPSS 22.0 software. We applied the factor analysis of the preference system as a first step in the segmentation according to food consumer preference, within which we determined the final factor structure based on the KMO value, total variance value, and professional explicability. We used a K-means clustering process to segment the data which is a statistically sound technique in samples larger than 1,000 items. In the present study, in addition to the results of factor and cluster analysis, we used Pearson’s Chi-square significance values to establish statistical correlations during segment characterization while the absolute values of Adjusted Residual (hereinafter Adj.R) were taken into account to establish and analyze internal correlations.

## Results and discussion

According to the main socio-demographic characteristics of the sample, 60% of the respondents were women and 40% were men. In terms of age, the highest proportion of respondents were aged 16–20 (31.1%), followed by those aged 21–25. (24.5%). In other words, more than half of the sample (55.5%) were respondents under 25 years old, i.e. Generation Z. Unsurprisingly, given the age, 42% of respondents were single and 54% were married or in a civil partnership. 42% of the respondents live in the capital, 38% live in a city and only 20% live in a village or hamlet. In terms of educational attainment, those with secondary education were absolutely over-represented (70%). To test our hypothesis, we segmented the sample for the first time according to the results of a factor analysis carried out on the grocery shopping preferences list. Our aim was to find out which factors form a unity in consumers’ value judgments of food purchase aspects. The factor analysis helped to reduce the number of food purchase criteria and the resulting factor structure provided the basis for clustering.

In the factor analysis, the principal component analysis method was used to select the number of factors, and the Varimax with Kaiser normalisation method was used to rotate the factors. The Kaiser-Meyer-Olkin criterion and the Bartlett test were used to assess the fitness of the data. Multiple rotations were carried out in the analysis, and results obtained for different factor scores were also evaluated relative to each other.

The four-component variant was the statistically and professionally best solution factor structure (Table 2).

- F1: The first factor is the ‘Design and Communication Elements’ group which includes elements such as packaging, marketing and functional features, brand name and advertising.
- F2: The ‘Origin and Content Values Group’ included taste and smell aspects and the place of food origin.
- F3: Purchasing factors related to discounts and promotions were included in the ‘Price Sensitivity’ factor.
- F4: The ‘Convenience Considerations and Information Elements’ factor group included durability and availability as well as the trademark as a purchasing preference element.

**Table 2:** Factor matrix of preference list in the case of food purchase.

Elements	Factors			
	F1 = Design and Communication Elements	F2 = Origin and Content Values Group	F3 = Price Sensitivity	F4 = Convenience Considerations and Information Elements
**Attractiveness of packaging**	0.745	0.016	0.146	-0.065
**Food advertising**	0.731	-0.005	0.079	-0.049
**Brandname**	0.619	0.065	-0.006	0.193
**Practicality of packaging**	0.602	0.215	0.027	0.261
**Geographical origin (place of origin of the food)**	0.100	0.866	0.016	0.000
**Food made exclusively from Hungarian ingredients**	0.293	0.756	-0.033	0.015
**Content values**	-0.188	0.533	0.140	0.191
**The food should be cheap**	0.046	-0.009	0.884	0.132
**Food should be on sale**	0.157	0.090	0.848	0.063
**Food durability, shelf life**	-0.050	0.066	0.071	0.819
**Be easily accessible**	0.169	0.019	0.213	0.714
**Includes a packaging trademark**	0.311	0.387	-0.206	0.494

Source: Own research, 2020 N = 1447, KMO = 0.697; total variance = 59.80%, Approx. Chi-Square: 2961.778; df = 66; sig = 0.00;

K-means was used to conduct cluster analysis on the resulting factor structure (Table 3). As a result, we were able to distinguish between the following food buyer segments, confirming our hypothesis H1:

- ‘Impulse Buyers’ (N = 408): those who purchase food based on its external, recognisable features, and commercials.
- As opposed to the other segments, ‘Conscious Food Buyers’ (N = 348) were the most likely to consider the category of factors of geographical elements and content values to be the most important.
- ‘Price Sensitive’ (N = 392): for whom the range of price-related elements, sales, and discounts are the most relevant criterion when selecting food.
- ‘Non-preferential’ (N = 299): those who buy food with an immature concept did not find any of the factor groups to be truly authoritative. Presumably, they are the consumers who do not yet have a mature value system. In many cases, they are more easily influenced, and the right knowledge can be brought to them through educational campaigns.

**Table 3:** Consumer segments formed on the basis of food purchasing preferences.

Factors	Consumer segments			
	Impulse Buyers N = 408	Conscious Food Buyers N = 348	Price Sensitive N = 392	Non-preferential N = 299
**Design and Communication Elements**	0.96648	-0.53918	-0.48289	-0.05817
**Origin and Content Values**	0.11948	1.15585	-0.67692	-0.62085
**Price Sensitivity**	-0.30098	0.04873	0.74282	-0.61988
**Convenience Considerations and Information Elements**	0.52225	-0.15207	0.43893	-1.11110

Source: Own research, 2020 N = 1447

To confirm the hypothesis, we used a segment-specific questionnaire to look at people’s views on Hungarian food and attitudes toward it.

According to Pearson’s Chi-square result, we were able to create a statistically verifiable correlation between judging subsequent statements and belonging to the food shopping segment (Table 4). The corrected standardized residual value was used to analyze the internal correlation (H2 confirmed).

**Table 4:** Opinions of food customer segments on the quality of Hungarian food.

Food customer segments		The quality of Hungarian food compared to normal food				Sum
		better	worse	same	I do not know	
**Impulse Buyers**	row%	42.6	7.4	38.7	11.3	100.0
	column%	30.4	36.6	27.2	21.7	28.2
	Adjusted Residual	1.5	1.7	-0.7	-2.3	
**Conscious Food Buyers**	row%	54.3	2.3	33.3	10.1	100.0
	column%	33.0	9.8	20.0	16.5	24.0
	Adjusted Residual	6.5	-3.1	-3.0	-2.8	
**Price Sentitive**	row%	26.0	5.9	47.2	20.9	100.0
	column%	17.8	28.0	31.8	38.7	27.1
	Adjusted Residual	-6.4	0.2	3.3	4.1	
**Non-preferential**	row%	35.8	7.0	40.8	16.4	100.0
	column%	18.7	25.6	21.0	23.1	20.7
	Adjusted Residual	-1.5	1.1	0.3	1.0	
**Sum**	row%	39.5	5.7	40.2	14.7	100.0
	column%	100.0	100.0	100.0	100.0	100.0

sig = 0.000

Source: Own research, 2020 N = 1447, measurement levels: nominal, attributes = clusters Chi-square test, Adjusted Residual = corrected standardized residues

In view of this, we can conclude that among the ‘*Conscious Food Buyers*’ the proportion of those who believe Hungarian food is of better quality is higher than predicted. In comparison, in the ‘*Price Sensitive’* group, this proportion was lower than expected but the proportion of those who believe there is no difference in quality between Hungarian and non-Hungarian food is higher.

We observed a similar disparity between the two segments when it came to the reliability of Hungarian food (Table 5).

**Table 5:** Opinions of food customer segments on the reliability of Hungarian food.

Food customer segments		Reliability of Hungatian food compared to normal food				Sum
		better	worse	same	I do not know	
**Impulse Buyers**	row%	39.7	5.6	43.4	11.3	100.0
	column%	29.8	30.7	27.8	23.8	28.2
	Adjusted Residual	1.1	0.5	-0.3	-1.4	
**Conscious Food Buyers**	row%	52.0	3.4	32.2	12.4	100.0
	column%	33.3	16.0	17.6	22.3	24.0
	Adjusted Residual	6.4	-1.7	-5.1	-0.6	
**Price Sentitive**	row%	26.3	4.6	53.6	15.6	100.0
	column%	19.0	24.0	33.0	31.6	27.1
	Adjusted Residual	-5.4	-0.6	4.5	1.5	
**Non-preferential**	row%	32.4	7.4	45.8	14.4	100.0
	column%	17.9	29.3	21.5	22.3	20.7
	Adjusted Residual	-2.0	1.9	0.7	0.6	
**Sum**	row%	37.5	5.2	44.0	13.3	100.0
	column%	100.0	100.0	100.0	100.0	100.0

sig = 0.000

Source: Own research, 2020 N = 1447, measurement levels: nominal, attributes = clusters Chi-square test, Adjusted Residual = corrected standardized residues

The proportion of those who thought Hungarian food was the most reliable was higher than predicted among the ‘*Conscious Food Buyers*’ while it was lower among the ‘*Price Sensitive*’.

In terms of the price of Hungarian food, we found that ‘*Impulse Buyers*’ did not perceive Hungarian food to be more expensive, whereas ‘*Conscious Buyers*’ believed Hungarian food to be less expensive in a lower proportion than predicted (Table 6). Those who found Hungarian food to be more costly, as well as those who claimed that these Hungarian goods could be purchased for a lower price, were categorized as ‘*Price Sensitive*’ and were fewer in number than expected.

**Table 6:** Opinion of food customer segments on the price of Hungarian food.

Food customer segments		The price of Hungarian food compared to normal food				
		higher	lower	same	I do not know	Sum
**Impulse Buyers**	row%	40.0	16.2	29.9	14.0	100.0
	column%	25.4	34.0	29.3	29.1	28.2
	Adjusted Residual	-2.1	1.9	0.6	0.3	
**Conscious Food Buyers**	row%	46.6	8.6	32.5	12.4	100.0
	column%	25.3	15.5	27.2	21.9	24.0
	Adjusted Residual	1.0	-3.0	1.8	-0.7	
**Price Sentitive**	row%	49.5	16.3	21.7	12.5	100.0
	column%	30.3	33.0	20.4	25.0	27.1
	Adjusted Residual	2.4	2.0	-3.6	-0.7	
**Non-preferential**	row%	40.8	11.4	32.1	15.7	100.0
	column%	19.0	17.5	23.1	24.0	20.7
	Adjusted Residual	-1.4	-1.2	1.4	1.2	
**Sum**	row%	44.3	13.4	28.7	13.5	100.0
	column%	100.0	100.0	100.0	100.0	100.0

sig = 0.001

Source: Own research, 2020 N = 1447, measurement levels: nominal, attributes = clusters Chi-square test, Adjusted Residual = corrected standardized residues

It is true that a higher proportion of those who want to buy Hungarian food with pleasure were reflected in both the ‘*Impulse Buyers*’ and the ‘*Conscious Customers*’ groups as this helps to sustain domestic workers (Table 7).

**Table 7:** Opinions of food purchasing segments on the job-creating ability of Hungarian foods in Hungary.

Food customer segments		I like to buy Hungarian food because, with this, I support Hungarian jobs		
		yes	no	Sum
**Impulse Buyers**	row%	80.6	19.4	100.0
	column%	30.2	22.1	28.2
	Adjusted Residual	3.0	-3.0	
**Conscious Food Buyers**	row%	90.5	9.5	100.0
	column%	28.9	9.2	24.0
	Adjusted Residual	7.6	-7.6	
**Price Sentitive**	row%	60.2	39.8	100.0
	column%	21.7	43.6	27.1
	Adjusted Residual	-8.1	8.1	
**Non-preferential**	row%	69.9	30.1	100.0
	column%	19.2	25.1	20.7
	Adjusted Residual	-2.4	2.4	
**Sum**	row%	75.3	24.7	100.0
	column%	100.0	100.0	100.0

sig = 0.000

Source: Own research, 2020 N = 1447, measurement levels: nominal, attributes = clusters Chi-square test, Adjusted Residual = corrected standardized residues

In the ‘*Non-Preferential*’ and ‘*Price Sensitive*’ segments, however, it was precisely those who did not tend to consider this incentive of satisfaction when buying Hungarian foodstuffs that were in a higher proportion than expected.

It is especially characteristic of ‘*Price Sensitive*’ to buy Hungarian food if the price is more favorable which is not a surprising result given the consumer preference of the given cluster while it is not explicitly typical of ‘*Conscious Customers*’ (Table 8).

**Table 8:** Opinions of food shopping segments on the purchase of cheaper Hungarian food.

Food customer segments		I only buy Hungarian food if it is cheaper than normal food		
		yes	no	sum
**Impulse Buyers**	row%	23.5	76.5	100.0
	column%	26.4	28.8	28.2
	Adjusted Residual	-0.9	0.9	
**Conscious Food Buyers**	row%	8.9	91.1	100.0
	column%	8.5	29.3	24.0
	Adjusted Residual	-8.0	8.0	
**Price Sentitive**	row%	40.8	59.2	100.0
	column%	44.0	21.4	27.1
	Adjusted Residual	8.4	-8.4	
**Non-preferential**	row%	25.8	74.2	100.0
	column%	21.2	20,.	20.7
	Adjusted Residual	0.3	-0.3	
**Sum**	row%	25.2	74.8	100.0
	column%	100.0	100.0	100.0

sig = 0.000

Source: Own research, 2020 N = 1447, measurement levels: nominal, attributes = clusters Chi-square test, Adjusted Residual = corrected standardized residues

The idea that ‘*Impulse Buyers*’ buy Hungarian food under the influence of their friends is particularly typical of them while ‘*Price Sensitive*’ people do not (Table 9).

**Table 9:** Purchasing Hungarian food under the influence of friends among food shopping segments.

Food customer segments		I buy Hungarian food because my friends buy it too		
		yes	no	Sum
**Impulse Buyers**	row%	12.3	87.7	100.0
	column%	36.2	27.3	28.2
	Adjusted Residual	2.2	-2.2	
**Conscious Food Buyers**	row%	9.8	90.2	100.0
	column%	24.6	24.0	24.0
	Adjusted Residual	0.2	-0.2	
**Price Sentitive**	row%	5.6	94.4	100.0
	column%	15.9	28.3	27.1
	Adjusted Residual	-3.1	3.1	
**Non-preferential**	row%	10.7	89.3	100.0
	column%	23.2	20.4	20.7
	Adjusted Residual	0.8	-0.8	
**Sum**	row%	9.5	90.5	100.0
	column%	100.0	100.0	100.0

sig = 0.012

Source: Own research, 2020 N = 1447, measurement levels: nominal, attributes = clusters Chi-square test, Adjusted Residual = corrected standardized residues

This further suggests that ‘*Impulse Buyers*’ are a quickly affected category that is particularly vulnerable to external impacts (stimuli, impressions).

The chic, trendy, characteristic of Hungarian food usually motivates ‘*Impulse Buyers*’ and, not surprisingly, those ‘*Non-Preferential’* with unstable beliefs and therefore can readily be persuaded to purchase it. This motivational influence is absent in the case of ‘*Price Sensitive Food Buyers*’ (Table 10).

**Table 10:** Purchasing Hungarian food as a result of fashion and trend among food shopping segments.

Food customer segments		I buy Hungarian food because it is fashionable and trendy		
		yes	no	Sum
**Impulse Buyers**	row%	4.9	95.1	100.0
	column%	41.7	27.7	28.2
	Adjusted Residual	2.1	-2.1	
**Conscious Food Buyers**	row%	2.0	98.0	100.0
	column%	14.6	24.4	24.0
	Adjusted Residual	-1.6	1.6	
**Price Sentitive**	row%	0.8	99.2	100.0
	column%	6.3	27.8	27.1
	Adjusted Residual	-3.3	3.3	
**Non-preferential**	row%	6.0	94.0	100.0
	column%	37.5	20.1	20.7
	Adjusted Residual	2.9	-2.9	
**Sum**	row%	3.3	96.7	100.0
	column%	100.0	100.0	100.0

sig = 0.012

Source: Own research, 2020 N = 1447, measurement levels: nominal, attributes = clusters Chi-square test, Adjusted Residual = corrected standardized residues

The results of previous surveys of Hungarian consumers show a generally positive perception of domestic products. The quality and reliability of domestic products were also positively assessed by respondents in our survey, thus the results of previous surveys on similar topics were in line with the opinion of our respondents [64–66]. Previous Hungarian research on ethnocentric behaviour in domestic food shopping has clearly demonstrated that consumers show cognitive dissonance in the conative, i.e. action, part. One of the main results of our research is that we have been able to identify possible food consumer segments with a potential for buying domestic products. Complementing the marketing strategy recommendations of previous research, we found that the use of targeted communication activities can best help encourage consumers to buy via education campaigns and engaging communication messages being the most effective.

## Conclusions

In the theoretical part of our study, we analyzed the impact of ethnocentrism on consumer behaviour and food consumption patterns based on the conclusions of relevant international research and domestic studies. We have presented food consumption trends in general, without going into detail, to provide an overview of the factors that may have a relevant impact on food consumption behaviour, including ethnocentric consumer behaviour.

In the course of the theoretical overview, different interpretations of ethnocentrism, the reasons behind its emergence and consumer motivations are presented. By comparing international and domestic studies, we have identified common points of intersection as well as differences. It was precisely the need for a more nuanced understanding of these differences that prompted the primary research. In this context, we analyzed the perception of domestic food in the context of food buyer preference, providing a new facet to ethnocentric consumer behaviour research.

Indeed, in the primary research, ethnocentric behaviour and how domestic food is perceived were analyzed along the lines of food buyer preferences, rather than along consumer socio-demographic and/or lifestyle characteristics, as was the case in most of the literature we analyzed. In the framework of independent primary research, we sought to discern which food consumer segments in our country could be potential buyers of domestic products, and how different food consumer groups relate to domestic products.

Overall, we confirmed our hypothesis that the opinions and attitudes of the food consumer segments—according to their food consumer preferences—differ with regard to Hungarian food. We performed a factor analysis for the factors of food buyer preferences with data reduction and segmented the sample based on the results.

The factor analysis allowed us to characterize four groups based on statistical and technical criteria: ’Design and Communication Elements’, ’Origin and Nutritional Values group’, ’Price Sensitivity’, and ’Convenience and Information Elements’.

As a result of the cluster analysis carried out on the factor groups, four distinct consumer segments could be identified: ‘Impulse Buyers’ (N = 408), who choose food products mainly on the basis of their external, visible elements and advertising. ‘Conscious Food Buyers" (N = 348), who are influenced by the geographical origin and the nutritional value of the food. ‘Price-sensitive’ (N = 392), for whom price and promotions were the most important factors. Finally, there is the ‘No Preference’ group (N = 299 persons), who did not rate any of the variables studied as important above average.

This was followed by an analysis of each segment’s perception of domestic food and their main reasons for buying it. According to the results, the quality and reliability of Hungarian food is the reason why ‘Conscious Food Buyers’ choose Hungarian food. This segment is considered the main consumer base for Hungarian food in light of the results.

In our opinion, ‘Impulse Buyers’ and ‘Those Without Preferences’ could be potential target groups for Hungarian food as a result of an education and communication campaign based on the right reference person and sufficiently fashionable and trendy motifs. These are the easily influenced segments with often still immature preferences and decision criteria who are not dominated by price sensitivity, and are therefore willing to pay a higher price for a product if it is fashionable, trendy and their friends accept the purchase result. They are more likely to be motivated by social recognition.

In our view, the ‘price-sensitive food buyer segment’ is not a potential target market for Hungarian food. In their case, price-related elements are so strongly driving their purchases that it is almost impossible or unprofitable to change this preference system. A practical adaptation of our research is provided by the results of segment characterization. We have identified the type of food buyers that can be considered as potential consumers of domestic food. We have also been able to identify the potential additional consumers who could be persuaded. In this respect, the results can help to position domestic food brands, indicating possible ways of expanding the target group. The results will also help to understand the reasons for consumers’ motivation to buy or not to buy domestic food products which can also provide practical support for the development of marketing activities.

One limitation of primary research is the local nature of the results due to sampling. The research did not take into account the variation in the place and type of residence of the sample. In our view, place of residence may also be a determinant of food purchasing habits and ethnocentric consumer behaviour, so we plan to continue the research to explore regional specificities, their impact on food purchasing preferences and ethnocentric food consumer behaviour and to change the sampling procedure accordingly.

In addition, we plan to continue the research by analyzing the impact of the pandemic on food purchasing behaviour and ethnocentric food purchasing behaviour. A further aspect of continuing the research is a repeat sampling at a later stage which could reveal not only which changes in food consumption and purchasing behaviour have become relevant in the wake of the pandemic, but whose impact extends beyond the pandemic period; changing the way consumers make decisions over time. In the continuation of our research, we will focus on examining the socio-demographic characteristics of each segment and on analyzing further affective components of their knowledge and attitudes towards Hungarian food. In our view, the results can provide Hungarian food producers and distributors with a basis for mapping potential domestic segments and characterizing potential market expansion opportunities.

## Supporting information

S1 Data (XLSX)
